This article has been retracted.

# The use of machine translation algorithm based on residual and LSTM neural network in translation teaching

**DOI:** 10.1371/journal.pone.0240663

**Published:** 2020-11-19

**Authors:** Beibei Ren

**Affiliations:** College of Translation Studies, Xi’an Fanyi University, Xi’an, China; University College London, UNITED KINGDOM

## Abstract

With the rapid development of big data and deep learning, breakthroughs have been made in phonetic and textual research, the two fundamental attributes of language. Language is an essential medium of information exchange in teaching activity. The aim is to promote the transformation of the training mode and content of translation major and the application of the translation service industry in various fields. Based on previous research, the SCN-LSTM (Skip Convolutional Network and Long Short Term Memory) translation model of deep learning neural network is constructed by learning and training the real dataset and the public PTB (Penn Treebank Dataset). The feasibility of the model’s performance, translation quality, and adaptability in practical teaching is analyzed to provide a theoretical basis for the research and application of the SCN-LSTM translation model in English teaching. The results show that the capability of the neural network for translation teaching is nearly one times higher than that of the traditional N-tuple translation model, and the fusion model performs much better than the single model, translation quality, and teaching effect. To be specific, the accuracy of the SCN-LSTM translation model based on deep learning neural network is 95.21%, the degree of translation confusion is reduced by 39.21% compared with that of the LSTM (Long Short Term Memory) model, and the adaptability is 0.4 times that of the N-tuple model. With the highest level of satisfaction in practical teaching evaluation, the SCN-LSTM translation model has achieved a favorable effect on the translation teaching of the English major. In summary, the performance and quality of the translation model are improved significantly by learning the language characteristics in translations by teachers and students, providing ideas for applying machine translation in professional translation teaching.

## 1. Introduction

As the trend of economic and cultural globalization continues to intensify, the demand for translation has increased dramatically [1]. Compared with human translation, machine translation has two sides. On the one hand, it is cheaper and faster. On the other hand, it has more errors and uncomfortable sentences. However, with the emergence of new technologies, the disadvantages of machine translation are declining [2]. People from all walks of life are using machine translation to improve office efficiency and quality. Machine translation is helping people to break the translation barriers in communication [3]. Machine translation was originally the translation based on a certain rule RBMT (Rule Based MT), developed to the example-based translation EBMT (Example Based MT), and to the statistical machine translation SMT (Statistical MT) in the 1990s. Now, it has entered the neural network machine translation NMT (Neural MT) stage [4]. The core of machine translation is to improve translation quality. Deep neural network has made great progress in speech recognition and image recognition, but have encountered difficulties in the field of natural translation processing [5]. Until 2016, Google launched the GNMT (Google Neural Machine Translation), a multilingual neural network machine translation system based on deep learning. Compared with Google’s previous phrase-based statistical machine translation system, the translation error rate has dropped by 60%, which is close to the level of human translation [6]. It can be seen that the application of neural network in machine translation has great difficulties, which requires further investigation.

After performance comparison testing, neural network machine translation is significantly better than phrase-based statistical machine translation. This conclusion has been confirmed by multiple investigations [7–9]. In the application of machine translation, some scholars have proposed that machine translation can be used in teaching. It can enhance students’ cognition of human translation and machine translation, and cultivate their ability to apply machine translation [10]. Yao (2017) found that more English teachers worldwide began to try to apply machine translation to the teaching process, but few applications in China [11]. A survey by Wu and Zhang (2018) showed that compared with traditional English teaching, students who use machine translation have a better understanding of the classroom and help to improve translation skills [12]. Omar and Gomaa (2020) found that when students encounter difficult vocabulary, structure, and pragmatics in the classroom, the use of machine translation will have a negative impact on the reliability of these translations [13]. Läubli and Green (2019) [14] pointed out that the role of human-computer interaction should be fully utilized. With the help of machine translation and computer-assisted translation, the correct method of use should be adopted to improve teaching interest, accuracy, and sustainability, reducing the misuse of after-school learning [14]. Thus, it can be seen that machine translation is widely used in professional translation teaching, but no scholars have proposed the application of neural network machine translation technology in translation teaching.

Based on previous works, N-tuples, neural network, fusion, and other translation models are constructed. Plenty of translated materials are used for learning. Different models are trained and tested on GodEye and PTB (Penn Treebank) data sets. Through the analysis of the model’s performance, translation quality, adaptability, and teaching evaluation, it is hoped to verify the advantages and disadvantages of the translation model based on SCN (Skip Convolutional Network) and LSTM (Long Short Term Memory) in teaching research applications. To a certain extent, it can promote the transformation of the translation talent training model and content, and accelerate the translation service industry to apply machine translation in the production process more widely and deeply.

## 2. Methods

### 2.1 Theoretical basis of translation

The translation model describes the inherent laws of natural translation mathematically. It is applied to various tasks requiring probabilistic evaluation of sentence sequences and is the key and cornerstone of text and speech signal processing. The function of the translation model is to calculate the probability that different words can form a sentence and to determine which word sequence is more likely to appear and to be spoken. Besides, the translation model can also predict the next most likely word based on the sequence of several words given. The acoustic model, the translation model, and the decoder constitute a complete speech recognition engine, and the translation model serves to evaluate the probability of all possible results decoded by the decoder. The sequence of words with the highest probability is the text recognized. The functional diagram of the specific translation model is shown in Fig 1.

**Fig 1:** Functions of a translation model.

Translation models with excellent presentation, comprehension, and calculation abilities have been trained continuously for academic and commercial purposes. The early translation model used in text and voice data processing mainly depends on writing grammar and syntactic rules manually. Due to the diversity and complexity of text and voice data, this rule-based approach is time-consuming and laborious and unable to cover complex translations. Besides, it has low robustness and requires the participation of translation experts. As a result, the rule-based approach cannot be widely used for its incapability of solving the core problems in translation. In the late 1980s, a translation model that could learn the inherent mathematical laws of translations in large corpora was constructed by combining statistics with computational translation studies. This model, with simple algorithms and easy implementation, is wide-accepted by the industry. However, the statistics-based translation model shows inferior performance in deep semantic understanding. Research on translation models has entered another stage with the introduction and successful application of artificial neural networks and deep neural networks. So far, the study of the translation model has gone through several stages, including a rule-based translation model, a statistic-based translation model, a feed-forward neural network translation model, and a deep neural network translation model.

### 2.2 Traditional machine-learning translation model

In machine translation, the most common translation model is N-tuple, which is widely used in traditional teaching. N-tuple is a statistical method calculating the probability model of sentences following translation logic [15], whose translation accuracy is low. The N-tuple translation model relies on the Markov hypothesis, which assumes the appearance of the next word in translation only depends on the finite number of words in front of it, leading to many problems in professionalism. The commonly used N-Tuple translation models include Bigram, Trigram, and four-gram [16]. The N-tuple translation model is usually constructed as the probability distribution of a word or word sequence, and its probability equation is:

P(S)=P(w1)*P(w2/w1)*P(w3/w1w2)*…*P(wn/w1…wn−1) (1)

Where: *w*_*i*_ represents a word in a sentence. *P*(*W*_*n*_/*W*1…*W*_*n*-1_) represents the probability of the sequence consisting of *w*_*1*_*…w*_*n*_ appearing as a sentence. In this method of probability calculation, as the word sequence increases, the complexity of the calculation will increase exponentially. It is assumed that the occurrence of each word in the text is only related to the previous *n-1*. In general, the value of *n* is not too large. Therefore, the calculation of the general binary translation model is as follows.

$$P(S)\approx P(w_{1})*P(w_{2}/w_{1})*P(w_{3}/w_{1}w_{2})*\ldots *P(w_{n}/w_{1}\ldots w_{n-1})$$ (2)

The calculation of the Trigram translation model is as follows.

$$P(S)\approx P(w_{1})*P(w_{2}/w_{1})*P(w_{3}/w_{1}w_{2})*\ldots *P(w_{n}/w_{\text{n}-2}w_{n-1})$$ (3)

The larger of the value of *n* in the N-tuple translation model, the more information obtained, the more accurate the prediction of the next word, the more the model parameters.

### 2.3 Construction of translation model based on neural network

(1) RNN (Recurrent Neural Networks) is the most commonly used ring structure network in machine learning. It can persist in data information and can learn data with time-series information. The translated text data is natural data with sequence information. Therefore, some researchers have proposed that RNN can be introduced into the investigation of translation models [17]. The structure diagram of a classic RNN is shown in Fig 2.

**Fig 2:** Structure diagram of RNN neural network.

According to the related investigation of machine translation and RNN [18], a specific RNN translation model is proposed, as shown in Fig 3. First, the pre-trained word vector is directly input into the network. A word vector is used to represent a word and is often considered the eigenvector of a word. Now, it has become the necessary technology of natural language processing. The quality of the word vector will directly affect the experimental results of the model. Without GPU resources, training word vectors is a time-consuming process, and word vectors trained are not necessarily good.

**Fig 3:** Construction of translation model based on RNN.

(2) CNN (Convolution Neural Network) is a neural network structure algorithm based on a multilayer perceptron. CNN can effectively learn semantic features and has been successfully applied in various fields [19]. It is generally composed of three parts: an input layer, output layer, and hidden layer. The greatly important one is the hidden layer, which includes weight sharing, local perception, and translation invariance. In a standard deep neural network, each neuron in the hidden layer is connected to the neurons in the adjacent layer one by one. It is difficult to analyze the connection between the two sentences during the translation process [20]. The local perception feature of CNN effectively avoids this connection. As shown in Fig 4, only a limited number of neurons are connected between each layer.

**Fig 4:** Schematic diagram of local perception based on CNN.

(3) SCN is inspired by the outstanding results of deep learning applications in computer vision and improvements of hardware computing power, which incorporates deep learning ideas. Traditional shallow learning can only manually extract features for simple function fitting; in contrast, deep learning can automatically learn the hierarchical features and approximate more complex nonlinear function models. The performance of SCN reconstruction based on deep learning surpasses that of many classical algorithms and becomes a research hotspot. Fig 5 shows the SCN structure.

**Fig 5:** SCN structure.

The SCN algorithm designs a CNN with two hidden layers and one output layer to learn the nonlinear mapping relationship between LR (Low Resolution) image block and HR (High Resolution) image block to predict HR image directly based on the LR image. The SR reconstruction algorithm based on sparse representation can also be regarded as a 3-layer neural network. SCN can reconstruct the whole image efficiently and effectively, and the network structure is simple and easy to converge. CNN will deepen the network without adding parameters, to learn the mapping model of LR image to HR image.

### 2.4 Construction of translation model based on fusion algorithm

As one of the variants of RNN, LSTM (Long Short Term Memory) has been successfully applied in text sequence modeling [21]. An LSTM unit contains an input gate, output gate, and forget gate. Among them, the input gate controls the input of the model, the output gate controls the output of the model, and the forget gate calculates the degree of forgetting of the memory module at the previous moment. The structure of the LSTM model is shown in Fig 6, and the specific calculation equation is as follows.

**Fig 6:** LSTM model structure diagram.

$$f_{t}=\sigma (W_{f}\cdot [h_{t-1},x_{t}]+b_{f}$$ (4)

$$i_{t}=\sigma (W_{\text{i}}\cdot [h_{t-1},x_{t}]+b_{\text{i}}$$ (5)

$$C=\tanh(W_{\text{c}}\cdot [h_{t-1},x_{t}]+b_{c}$$ (6)

$$C_{\text{t}}=f_{t}\times C_{t-1}+i_{t}\times C$$ (7)

Where: *f*_*t*_ and i_*t*_ respectively represent the forget gate and the input gate at the step *t* in the sentence sequence. In each sentence sequence, the forget gate controls the degree of forgetting the information of each word, and the input gate controls the degree to which each word information is newly written into long-term information. The two gates of *f*_*t*_ and i_*t*_ use the Sigmoid function. The range of the value is [0,1] and the value of the tanh function is [–1,1]. *C*_*t*-1_is the state of the neuron at time *t-1*., *C*_*t*_ is the state of the neuron at time *t*.

$$h_{t}=o_{t}\times \tanh(C_{t})$$ (8)

$$o_{t}=\sigma (w_{o}\cdot [h_{t-1},x_{t}]+b_{o}$$ (9)

Where: *o*_*t*_ is the output degree of the output gate controlling word long-term information. *h*_*t*_ is the output of step *t* in the sentence sequence. From the equation, it can be known that the word information of the current step of LSTM is determined by the word information retained in the previous step and the word information saved after being filtered by the input gate at the current time.

The application of the LSTM model in translation has the problem of insufficient learning and training. SCN is a kind of CNN, which can effectively analyze different sentences [22]. Based on this, the SCN-LSTM (Skip Convolutional Network and Long Short Term Memory) fusion translation model is proposed. The specific structure is shown in Fig 7. The feature extractor uses SNN and LSTM respectively. The model contains three convolutional layers and two LSTM layers to extract text features. In the convolutional layer part, the skip connection convolution structure (SCN) is adopted. In the second half of the model, the merge layer is used to merge the word vectors of the SCN and the input layer. First, the expanding reshape operation is performed on the output of the SCN layer. The dimension is adjusted to the same dimension as the input layer subsequence. The specific operations of the merge layer include point-by-point addition and multiplication of vectors and direct vector splicing. In this investigation, the point-by-point addition of vectors is selected. Specifically, the output of the SCN layer is sent to the expansion layer for data dimension alignment. Then, it adds point by point to the sentence vector of the input layer. After merging the layers, the encoded information is input to the LSTM layer. The LSTM layer includes two layers of LSTM, and the LSTM layer is connected to the Softmax layer. In the Softmax layer, the output of the LSTM layer is connected to a fully connected layer, and Softmax operation is performed on it.

**Fig 7:** Construction of translation model based on SCN-LSTM.

### 2.5 Other neural network translation models

To prove the effectiveness of the model proposed, many translation models implemented by different mainstream text feature extractors are trained and tested, namely GRU (Gated Recurrent Unit) translation model, LSTM translation model, and CNN-LSTM translation model. The data preprocessing process is the same as the SCN-LSTM model. The specific model topology is shown in Figs 8 and 9, respectively.

**Fig 8:** GRU and LSTM translation models.

**Fig 9:** GNN-LSTM translation model.

### 2.6 Algorithm data set and model training

1. Dataset: the data used here mainly comes from two sources. One is the *College Professional English* textbook. Its electronic content is found and is marked as GodEye. Due to its large amount, part of the text is deleted, and the rest is manually transcribed and segmented for inputting into the model. The other is the public PTB dataset. PTB is the most widely used dataset in language model learning and is commonly used to train RNN as language prediction [23]. TensorFlow also defines its function library for reading the PTB dataset. The models file in Python can be directly imported into the PTB library function to invoke further the dataset, where the ratio of the training set versus the test set is 8:2.
2. Model training: On the experimental machine, 8 Nvidia V100 series GPU graphics cards are used to train the network. For text data, it is necessary to remove punctuation and other special symbols. After getting the cleaned data, the word embedding model is trained. After being converted into a word vector, it can be applied to various deep neural network structures. A sentence is evenly segmented. On the GodEye data set, the average length of the text is 14.63. Therefore, 15 will be used as a subsequence length for segmentation. In the SCN feature extractor, ReLU is selected as the activation function. Each convolutional layer in the SCN layer is set with 8 convolution kernels. The first layer convolution kernel size is 7, the second layer convolution kernel size is 5, and the third layer convolution kernel size is 3. The sliding steps of the convolution kernels of the three convolutional layers are all 1. The number of neurons in the two-layer LSTM is 256. The output dimension of Softmax is 10000. The weight initialization of the model is a random initialization of truncated normal distribution.

### 2.7 Translation quality, model performance, and teaching evaluation

(1) Translation quality evaluation: confusion degree is the optional scope of the next possible word for any given word sequence [24]. The lower the confusion degree, the better the performance of the translation model. The fundamental step of getting the confusion degree is to calculate relative entropy, which measures the degree of closeness between two probability distributions. The definitions of entropy, cross entropy, and relative entropy are as follows.

$$/H(p)=-\sum_{i}p(x_{i})\log\;p(x_{i})$$ (10)

$$H(p,q)=-\sum_{i}p(x_{i})\log\;\text{q}(x_{i})$$ (11)

$$D(p\|q)H(p,q)-H(p)=-\sum_{i}p(x_{i})\log p(x_{i})/\text{q}(x_{i})$$ (12)

Where: *p(x)* and *q(x)* are all modelings of random variable distribution. It is assumed that *p(x)* is the true distribution of the data, and *q(x)* is the distribution modeled for it. Because the entropy *Hp(x)* of the true data distribution is determined, the average cross entropy can be calculated after optimizing the relative entropy as follows.

$$H(S)=-\frac{1}{N}\log\text{p(}w_{1}\text{,}w_{2}\ldots w_{N}\text{)}$$ (13)

It can be seen from the equation that the smaller the cross entropy, the closer the probability distribution of the model is to the real data distribution. Cross entropy describes the average code length. On this basis, the translation perplexity PPL (Perplexity) can be obtained, and the calculation process is as follows.

$$\text{pr}\;elexity(S)=2^{H(s)}$$ (14)

To facilitate the calculation, the exponent is often used.

$$\text{pr}\;elexity(S)=2^{H(s)}=\sqrt[{N}]{1-p(w_{1},w_{2}\ldots W_{N})}$$ (15)

$$\text{pr}\;elexity(S)=2^{H(s)}=e^{H(S)}$$ (16)

(2) Model performance evaluation index: Pre (Precision) indicates the proportion of processed samples that are correctly classified as positive samples. Rec (Recall) represents the proportion of positive samples in the original positive samples. The F-value is a comprehensive evaluation index of the Pre and Rec of the model. MS (Matching Speed) indicates the time from data input to translation completion [25]. The specific calculation is shown below.

Rec=CN (17)

$$\text{pr}\;\text{e}=\frac{C}{C+E}$$ (18)

$$F-\text{value}=\frac{2\times P\times R}{P+R}$$ (19)

Where: N represents the number of manually labeled segmented words, E is the number of words incorrectly labeled by the word segmentation tool, and C is the number of words correctly labeled by the word segmentation tool.

(3) Model adaptability: it evaluates the most stable value using the confusion degree. Teaching evaluation is to apply different models in actual teaching and evaluate the feedback on teaching effect (questionnaire method). The same students (n = 50) are taught in different ways to avoid the influence of divergence among different students on evaluation results, and their feedbacks are collected immediately after every class (45min). The evaluation consists of teaching comprehension and teaching satisfaction. The former includes improving translation ability, the digestion of knowledge, the use of machine translation, and the differences from direct face-to-face teaching, and the latter includes adaptability, comfort, and necessity of machine learning methods. The results are classified as four dimensions: very satisfied, satisfied, average, and not good. The statistical method is utilized in testing reliability and attaining consequence. A total of 300 questionnaires were issued, and 269 were returned, with a response rate of 89.67%.

## 3. Results and discussion

### 3.1 Performance evaluation of machine translation model of neural network based on residual and LSTM

Fig 10 shows the performance difference of different neural network machine translation models in accuracy and recall rate. In terms of accuracy, comparing the GodEye and PTB data sets, the accuracy on the test set is lower than the training set. On GodEye, the accuracy of the model after learning is lower than that of the PTB professional data set learning. Among the translation models, the highest accuracy is the SCN-LSTM model, with an average accuracy of 95.21%. The second is the CNN-LSTM model, with an accuracy of 93.64%. Among the single models, the highest accuracy is the LSTM model, and the worst accuracy is the N-tuple model, with an average accuracy of only 81.34%. In terms of recall rate, the data trained by the PTB data set is significantly better than the GodEye data set. The largest recall rate is the SCN-LSTM model, with an average recall rate of 95.11%. The worst is still the N-tuple model, with an average recall rate of only 81.47%. The machine translation model of neural network based on residual and LSTM is superior to other models in accuracy and recall rate.

**Fig 10:** Evaluation of accuracy and recall rate of machine translation model of neural network based on residual and LSTM. Note: GodEye-1 is the training set on GodEye data, GodEye-2 is the test set on GodEye data, PTB-1 is the training set on PTB data, PTB-2 is the test set on PTB data, CNN-L is CNN-LSTM, SCN-L is SCN-LSTM model.

Fig 11 shows the performance difference of the F value and processing time of different neural network machine translation models. In terms of comprehensiveness, comparing the GodEye and PTB data sets, the F value is not much different. Also, the highest comprehensive evaluation is the SCN-LSTM model, with an average of 95.89%%. The worst accuracy is the N-tuple model, with an average of 81.34%. In terms of processing time, the results of the PTB data set test are obviously higher than the GodEye test data set. The shortest processing time is the N-tuple model, with an average processing time of 1.34ms. The longest time-consuming is the LSTM model, with an average time-consuming of 5.47ms. The above results indicate that the SCN-LSTM translation model is superior to other models in terms of comprehensiveness, while the N-tuple model takes the shortest time.

**Fig 11:** Evaluation of machine translation model of neural network based on residual and LSTM in F value and processing time.

### 3.2 Evaluation of machine translation model of neural network based on residual and LSTM in translation quality

As shown in Fig 12, the results on different test sets show that, compared with the N-tuple model, the perplexity of the RNN translation model is reduced by 7.543 and the test set is reduced by 10.2%. Because the RNN translation model can learn a longer distance word sequence than the N-tuple translation model, it improves the performance of the translation model to a certain extent. However, the problems of the RNN translation model that cannot be trained in parallel and the gradient disappears during the training process have a serious impact on the training of the translation model. LSTM, one of the improved RNN, directly propagates backwards by adding intermediate state information, which effectively alleviates the problem of gradient disappearance and obtains better results. As can be seen from the above figure, the performance of the GRU translation model is not much different from the LSTM translation model. The simple superimposed convolutional layer model is difficult to converge and the model performance is difficult to improve. The combination of SCN, CNN, and LSTM greatly reduces the perplexity of the translation model. However, the model has a large difference between the test set and the training set. The phenomenon of model overfitting occurs. In summary, compared to other translation models, the translation quality of the combined approach is better.

**Fig 12:** Evaluation of translation quality of machine translation models based on deep learning neural networks.

### 3.3 Adaptability evaluation of machine translation model of neural network based on residual and LSTM

It can be seen from Table 1 that the performance of the fusion model is better than that of the single model. On the PTB data set, the adaptability of each translation model is lower than the GodEye data set, and the overall adaptability of the test set is lower than the training set. The reason is that GodEye is biased towards practical teaching applications, and the test set involves a small amount of data. Therefore, the model learning effect is better. The SCN-LSTM model has the best adaptability, which is 0.4 times that of the N-tuple model. In summary, the SCN-LSTM model can be better applied in actual teaching.

**Table 1:** Adaptability evaluation of machine translation model of neural network based on residual and LSTM.

Model	GodEye		PTB		Overview
	Training set	Test set	Training set	Test set	
N-tuple	60.903	61.34	62.56	64.58	62.34575
RNN	53.36	54.55	58.95	60.24	56.775
LSTM	49.56	51.22	53.12	55.36	52.315
GRU	51.23	53.59	53.56	58.47	54.2125
SCN-LSTM	37.45	40.12	41.76	43.59	40.73
CNN-LSTM	42.31	48.68	49.35	52.11	48.1125

### 3.4 Evaluation of machine translation model of neural network based on residual and LSTM in teaching application

Fig 13 illustrates the results of the actual teaching evaluations. Students using and not using machine translation are randomly selected for analysis. When not using machine translation technology, the classroom feedback is unfavorable, the students are more difficult to understand English, and their processing speed and acceptance of translation are slow. When using N-tuple machine translation based on sentence length and specific rules only, the students’ satisfaction and comprehension are generally low, 11%, and 27%, respectively. Such satisfaction and understanding of the machine translation model are significantly improved when the neural network is utilized, and the satisfaction of the fusion model is the highest. Many studies have reported that the neural network can improve translation quality; however, the neural network model is seldom used in English teaching. While results show significant advantages of the proposed teaching model. The SCN-LSTM machine translation model constructed gains a high degree of satisfaction and improves class comprehension, which can be used as an auxiliary teaching device to help students understand and learn English well.

**Fig 13:** Evaluation of machine translation model of neural network based on residual and LSTM in teaching application.

## 4. Conclusion

The shortcomings of the current translation model and its application in teaching are analyzed, and a machine translation model of neural network based on residual and LSTM is constructed. The addition of residual neural network can effectively improve the translation efficiency, LSTM effectively solves the convergence problem of neural networks in translation applications by adding intermediate state information to directly propagate backwards. Compared with other translation models on public translation data sets and actual data sets, it is found that the fusion model has better performance, translation quality, and teaching effect than the single model. The SCN-LSTM model has good generalization, and learns the language features of teacher and student translation well, so that the performance of the translation model is further improved. Although new models have been constructed and applied, there are still many shortcomings in the text: (1) The quantity and quality of the English training corpus designed in this investigation are poor. Therefore, the effect on the data set is significantly lower than the public data set. (2) The current investigation of translation models focuses on English. The Chinese-oriented investigation mostly draws on algorithms and ideas for English models. There is a big difference between Chinese and English. Chinese is an ideographic character that evolved from hieroglyphics. Therefore, how to use the font as a feature to join the translation model will be the focus of the next stage of the investigation.

## Supporting information

S1 Data (RAR)
